# Rationale and Criteria for a COVID-19 Model Framework

This article has been retracted.

**DOI:** 10.3390/v13071309

**Published:** 2021-07-06

**Authors:** Francesco Messina, Chiara Montaldo, Isabella Abbate, Manuela Antonioli, Veronica Bordoni, Giulia Matusali, Alessandra Sacchi, Emanuela Giombini, Gian Maria Fimia, Mauro Piacentini, Maria Rosaria Capobianchi, Francesco Nicola Lauria, Giuseppe Ippolito, on behalf of COVID-19 Scoping Review Working Group

**Affiliations:** 1 National Institute for Infectious Diseases, “Lazzaro Spallanzani”–IRCCS, Via Portuense, 292, 00149 Rome, Italy; francesco.messina@inmi.it (F.M.); chiara.montaldo@inmi.it (C.M.); isabella.abbate@inmi.it (I.A.); manuela.antonioli@inmi.it (M.A.); veronica.bordoni@inmi.it (V.B.); giulia.matusali@inmi.it (G.M.); alessandra.sacchi@inmi.it (A.S.); emanuela.giombini@inmi.it (E.G.); gianmaria.fimia@inmi.it (G.M.F.); mauro.piacentini@uniroma2.it (M.P.); maria.capobianchi@inmi.it (M.R.C.); francesco.lauria@inmi.it (F.N.L.); 2 Department of Molecular Medicine, Sapienza University of Rome, 00185 Rome, Italy; 3 Department of Biology, University of Rome Tor Vergata, Via della Ricerca Scientifica 1, 00133 Rome, Italy

**Keywords:** disease model, infectious disease systems, COVID-19, SARS-CoV-2 infections

## Abstract

Complex systems are inherently multilevel and multiscale systems. The infectious disease system is considered a complex system resulting from the interaction between three sub-systems (host, pathogen, and environment) organized into a hierarchical structure, ranging from the cellular to the macro-ecosystem level, with multiscales. Therefore, to describe infectious disease phenomena that change through time and space and at different scales, we built a model framework where infectious disease must be considered the set of biological responses of human hosts to pathogens, with biological pathways shared with other pathologies in an ecological interaction context. In this paper, we aimed to design a framework for building a disease model for COVID-19 based on current literature evidence. The model was set up by identifying the molecular pathophysiology related to the COVID-19 phenotypes, collecting the mechanistic knowledge scattered across scientific literature and bioinformatic databases, and integrating it using a logical/conceptual model systems biology. The model framework building process began from the results of a domain-based literature review regarding a multiomics approach to COVID-19. This evidence allowed us to define a framework of COVID-19 conceptual model and to report all concepts in a multilevel and multiscale structure. The same interdisciplinary working groups that carried out the scoping review were involved. The conclusive result is a conceptual method to design multiscale models of infectious diseases. The methodology, applied in this paper, is a set of partially ordered research and development activities that result in a COVID-19 multiscale model.

## 1. Introduction

To construct a large-scale comprehensive view of biological systems, several smaller models may need to be integrated. However, this can be difficult to accomplish, as models can exhibit significant inner variation due to the different expertise of modelers or perspectives of model.

Infectious disease modeling is an expansive field with a long history, encompassing a range of methods and assumptions that are not necessarily comparable or even designed for the same purpose. During the ongoing COVID-19 pandemic, the scientific community consider computer modeling as a possible solving factor given the enormous uncertainty about the evolution of the pandemic. In this context, epidemiological models can be critical planning tools for policymakers, clinicians, and public health practitioners [1]. Currently, COVID-19 modeling studies follow one of two general approaches: forecasting models and mechanistic models. However, these well-constructed statistical frameworks have several limits. These can be used for short-term forecasts through machine learning or regression to crunch past epidemiological data or data from different locations to make projections for the future [2].

Traditionally, the study of infectious disease systems was based on two main theories: infectious disease causation theory and infectious disease transmission theory.

The infectious disease causation theory incudes series of theories progressively refined, one after another as new knowledge, to explain the causes of infectious diseases and considers the infectious disease as systems [3]. The current and modern infectious disease causation theory considers infectious disease systems organized into hierarchical multilevel and multiscale complex systems, with levels ranging from cellular to macroecosystem one. The infectious disease transmission mechanism theory, instead, is based on the idea that infectious disease dynamics consist of transmission as main dynamic process at each hierarchical level (cell, tissue, host, etc.). Specific transmission models can be developed to study an infectious disease system at a particular level of organization. The standard approach to developing such models is to classify the reference population (may be population of cells at cell level or a population of hosts for the host level, and so on) into compartments within unit exanimated (cells, hosts, etc.). The knowledge about transmission mechanisms allows to develop quantitative models of infectious disease dynamics [4,5].

However, an infectious disease system is also result of the interaction of three subsystems (host, pathogen, and environment) organized into hierarchical multilevel and multiscale complex systems, with levels ranging from the cellular level to the macro-ecosystem level. The subsystems are decomposed into levels and then into scales. Therefore, to describe the phenomenon of infectious disease both in time and in space, it needs to define a model, where infectious disease systems are identified as multilevel and multiscale systems [5,6].

Recent advances in systems biology spawned the view of human disease as a manifestation of genetic and environmental perturbations to the human interactome, a key postulate being that similar perturbation patterns lead to similar disease phenotypes [7]. However, infectious diseases are extremely complex, as the dynamics of infection into the host could be influenced by the pathogen and the host response could induce adaptation events into the pathogen [8,9].

Computational modeling can contribute to a deeper understanding of relevant chemical and biological phenomena based on their underlying mechanisms, applying network-based model of viral–host interaction [10,11,12]. Simulations of models can help investigating a complete biological process instead of considering smaller segments or aspects, detailing a segment of a process. Moreover, data-driven inferences could suggest or even address future experiments, predicting with high statistical significance the behavior of system under given conditions and identifying unknown causal relationships from observational time series data [13].

Disease maps are an emerging concept, bridging bioinformatics, molecular biology, and clinical research, with the potential to link the domains of biomedical knowledge and data, providing an intermediate step between a conceptual and an executable model [14,15]. Such representation is an important tool to capture not only biochemical interactions, but also physiological mechanisms, describing the complexity of disease.

Previously, we carried out a scoping review of the literature based on conceptual domains to understand the molecular pathophysiology linking SARS-CoV-2 infection to its clinical manifestations (Montaldo and colleagues).

Thus, the further aim of our research group was to use the results of this scoping review along with other data from literature to design a multilevel and multiscale model framework for COVID-19. For this aim, at first a conceptual framework was built based on current literature evidence following these steps: to identify the molecular pathophysiology related to the clinical manifestations and course of COVID-19; to collect the mechanistic knowledge scattered across the scientific literature and bioinformatic databases; to integrate it using a logical/conceptual model systems biology. In the future, we will expect to assess the model in decision support.

In summary, here we describe the process and the methodology followed to build the modular design and conceptual framework of disease model for COVID-19.

## 2. Materials and Methods

The model building process began from building a domain-based literature review regarding a multi omics approach to COVID-19 (Montaldo and colleagues: Multiomics approach to COVID-19: a domain-based literature review). The results of this review allowed to define and validate a conceptual framework for COVID-19, representing these results on a multilevel and multiscale model.

The same interdisciplinary working groups that carried out the scoping review were involved for this purpose.

### 2.1. Step-by-Step Workflow for a Conceptual Framework of Disease Model

The conceptual framework for disease model of COVID-19 was designed investigating mainly interacting subsystems of host and pathogen. Such framework must be based on standard evidence derived from literature, appropriately identified and reviewed by domain-expert group. We carried out also a short literature review concerning methods, principles, and referral concept on infectious diseases modeling.

This methodological review, which we will call “short review”, is distinct from COVID-19 domain-based scoping review. The results of the short review are extensively reported in Supplement text.

To define the framework of this COVID-19 model, we followed the steps described below.

#### 2.1.1. Step 1: Multiomics Approach and Domains Identification Literature-Based

A conceptual model of a disease must contain disease-related signaling and metabolic and gene regulatory processes, with evidence of their relationships to pathophysiological causes and outcomes.

Therefore, it is necessary to develop and exploit protocols for high-quality representation of multilevel and multiscale information, including subcellular, cellular, tissue, organ, and organism levels.

Such amount of literature information must be reviewed and sorted by domain-expert group.

For this purpose, we assumed as conceptual reference the same studies, which were used to identify the conceptual domains on which our previous scoping review was based:

- Gordon and colleagues [16], which highlights interactions between SARS-CoV-2 proteins and human proteins involved in several complexes and biological processes, and multiple innate immune pathways involvement.
- Ostaszewski and colleagues [17,18]. The COVID-19 Disease Map is an open-access collection of curated computational diagrams and models of molecular mechanisms implicated in the disease.

Moreover, we consider the domain-based scoping review results, as reported in separated paper (Montaldo and colleagues). This scoping review is based on four conceptual domains (virus characterization, host signature, pathways and phenotypes) addressed within a disease network model. The results can be summarized as follows:

- the interactome method (as conceptually defined by Gordon and colleagues) is helpful to study the biology of the viral–host interactions and the biochemical pathways involved;
- the disease progression is mediated by commonly dysregulated pathways of innate immune responses, such as complement activation, inflammatory responses, neutrophil activation and degranulation, platelet degranulation, and dysregulation of blood coagulation and metabolism.

Table 1 reports the scoping review results detailed, aggregated in domains, and divided in subdomains.

Such results were especially useful in evaluating host response and identifying clinical COVID-19 phenotypes and could contribute to elaborate omics-based disease maps.

#### 2.1.2. Step 2: Defining Criteria and Framework for the COVID-19 Disease Model

To define criteria useful to building a logical model disease framework, we considered the following studies, which were more extensively reported in Supplement text:

Wong and colleagues (2020) [19]. A multiscale tissue simulator developed by an international and multi-disciplinary coalition, which could be used to investigate mechanisms of intracellular viral replication, infection of epithelial cells, host immune response, and tissue damage. It is a prototype of multiscale model of SARS-CoV-2 dynamics in lung tissue iteratively refined. To build the simulator, a modular design was used: an overall tissue-scale model integrates an array of targeted submodels that simulate critical processes (e.g., receptor binding and trafficking and virus replication). Each submodel is clearly specified to enable interoperability and to allow subteams to simultaneously develop and test the model components in parallel.

Perfetto and colleagues (2020) [20]. A dataset of physical molecular interactions, manually extracted by IMEx Consortium curators from 86 publications, focused on proteins from SARS-CoV-2, SARS-CoV and other members of the Coronaviridae family, currently comprises over 2,200 binarized interactions. Data on 70 organisms are included, and most interactions refer to SARS-CoV-2 and SARS-CoV-human host.

By these studies, we deduced that, to define the biological keys of COVID-19 model, these are the main criteria to follow:

(a) to investigate SARS-CoV2 dynamics;
(b) to help the scientific community to identify knowledge gap and to guide specific experiments and interventions (“what if …”);
(c) to be based on a modular design, where each module is divided into one or more submodules;
(d) one or more functions refer to submodules.

The same working groups that previously carried out COVID-19 domain-based scoping review compared the modular design, as above defined, to the results of this review, underlying a direct correspondence between module and domain.

Applying main criteria above reported to define the biological keys of the COVID-19 model, the following critical components of the model framework were identified:

- general model framework;
- module (tissue/organ and/or physiopathological mechanism);
- submodules that simulate critical process (receptor binding, cleavage and processing viral proteins, virus replication).

#### 2.1.3. Step 3: Normalization of the Biological Model on the Hierarchical Model

In the previous steps, we collected the mechanistic knowledge scattered across scientific literature and bioinformatic databases and integrated it using a logical/conceptual model systems biology. A model should also allow a correlation among host, pathogen, and environment.

For this step, we referenced results of the short review: principles and referral concepts for modeling of infectious diseases. An extensive description of results of the short review was reported in Supplement text. The aim was to identify through this short review a model framework that allows to describe infectious disease phenomena, considering possible variations through time and space at different scales. We identified methodology proposed by Garira, which incorporates events, such as pathogen replication, giving rise to transmission events in time and space. This methodology assumes that there are seven levels (cell, tissue, organ, microsystem, host, community, macrosystem), and within each level, there are two limiting adjacent scales of infection: microscale and macroscale. These levels hierarchically organized and make infectious disease dynamics at each level as a multiscale loop, involving the reciprocal influence of macroscale and microscale [4,5].

The main topics for building a disease model framework were:

- at any level of an infectious disease system, there is no privileged/absolute scale, which would determine disease dynamics, but only interactions between microscale and macroscale;
- at every level of an infectious disease system, the reciprocal influence between microscale and macroscale establishes a pathogen replication-transmission multiscale cycle;
- to use the conceptual diagram of the seven hierarchical levels of organization of an infectious disease system and the associated macroscale and microscale for each hierarchical level [21].

Here, we performed an alignment between multiscale levels and modules/domains as biologically defined above, considering the results of the literature review. We attributed a hierarchical scale among levels, and we associated macroscale/microscale for each level. The hierarchical scale macro/micro was defined considering module/submodule/functions, as organized in biological models reported above, and assuming that domain is assimilated into the module.

At last, we verified if the model framework is compliant with reciprocal influence between macroscale and microscale, types of environmentally transmitted infectious disease, following the Garira method, which was suitably adapted.

## 3. Results

Considering domains and datasets above identified and scoping review results, the following issues were considered useful to build a logical disease model framework:

- Virus dissemination in epithelial tissue;
- Virus binding, endocytosis, replication, and exocytosis;
- Infected cell responses: changes of metabolism, secreted signals, death;
- Inflammatory response;
- Ramp up of the immune response (particularly in lymph nodes);
- Immune cell infiltration;
- Immune cell predation of infected and other cells;
- Tissue damage by death of cells due to infection or host response.

We therefore performed the modular design of the COVID-19 model framework, biologically based. The logical process was an overall tissue-scale model that integrates an array of submodels, which simulate critical processes. Each submodel is clearly specified to enable interoperability and to allow subteams to simultaneously develop and test the model components in parallel. As expected in methods, the working group that previously carried out the COVID-19 domain-based scoping review translated the results of this review into modular logic (module/submodule/functions) of this model framework, as below reported:

- Module A: cell infection and viral replication (submodules: tissue microenviroment; binding receptor on the cell’s membrane (ACE2 system); endocytosis process; viral replication; assembled virions exported from the cell by exocytosis);
- Module B: infected cell response (submodules: activation IFN type1 signal; cell death process);
- Module C: inflammatory and immune responses (submodules: pneumocytes and alveolar macrophages; innate immune response; endothelial damage and systemic; tissue damage and cytokines);
- Module D: inflammatory and clinical outcomes (phenotypes), (submodules: dysregulated amplified immune response and chemokines replications in the lower airways persistence; systemic disease: interactions of viral infection, cytokine production, immune response; clinical syndromes: haemophagocytosis, intravascular coagulation, ARDS, organ failure).

The modular logic of the biological model framework is detailed in Table 2.

The main information about COVID-19 and SARS-CoV-2 infection were classified in four modules: cell infection and viral replication; infected cell response; inflammatory, adaptive, and innate immune responses; inflammatory, clinical outcome and phenotypes.

This setting, composed by module and submodules, allows to highlight multiple biological pathways in cells, tissues, organs, and define different COVID-19 phenotypes. However, this structure can provide a modular and ordered literature data but it cannot represent a framework for disease model, as levels (different point of view) and scales (within or between objects of analysis) are not provided.

Then, to consider possible variations at different scales for many levels, we first identified the macro/microscale attributions depending on the considered level, applying method logic of Garira.

Secondly, we considered the types of reciprocal influence among macroscale, microscale, and environment related to SARS-CoV-2 infection processes.

The Garira methodology assumes that the microscale and the macroscale influence each other at each hierarchical level of an infectious disease system through interactions of four key disease processes:

- infection/superinfection by pathogen;
- pathogen replication;
- pathogen shedding/excretion;
- pathogen transmission.

At each hierarchical level, disease dynamics involve a pathogen replication-transmission multiscale cycle. This happens because, at each of the hierarchical levels of organization of an infectious disease system, the characteristic scale at which pathogen replication and pathogen transmission occur often does not match.

Consequently, we distinguished two kinds of reciprocal influences between microscale and macroscale:

Type I: the microscale influences the macroscale through pathogen shedding/excretion: this involves the movement of pathogen from the microscale to the macroscale.

Type II: the macroscale influences the microscale also through super-infection.

(i.e., repeated infection before the host recovers from an infectious episode).

This condition involves the movement of the pathogen from the macroscale to the microscale. [5].

Furthermore, following the logic of Garira method, considering host as unit exanimated, it was possible to identify three different types of environmentally transmitted infectious disease systems: Type A, where the pathogen does not replicate within-host (microscale); Type B, where the pathogen replicates only within-host (microscale); Type C, where the pathogen replicates both within-host and between-hosts (microscale and macroscale).

An extensive description of the methodology regarding the mutual influence between micro/macroscale and the types of environmentally transmitted infectious disease systems are reported in Supplement text. Conceptual representation of mutual macro/micro scale influences and infections environmentally transmitted are in Table S1.

As descripted in methods, the biological model framework was normalized on the hierarchical model, appropriately adapted following Garira methodology, as below reported:

- Level from I to V:
  - Cell level: module A and module B. Cell infection and viral replication and infected cell response;
  - Tissue level: module C. Inflammatory, innate, and adaptive immune response;
  - Organ/anatomical compartment level: module C + D. Inflammatory, innate, and adaptive immune response;
  - Microsystem level: module C + B + A. The three previous modules can contribute to describe functional interactions between human host and multi pathogens, both within and between specific anatomical districts;
  - Host/organism level: module D + A. Inflammatory and clinical outcome, and phenotypes of host, transmission risk in hospital and family; social distancing;
- Level VI and VII:
  VI. Community level: epidemiological enquiries within community (familiar and hospital clusters, etc.) and between communities (restriction movement, etc.), global surveillance of infectious diseases;
  VII. Macrosystem level: dynamics of functional interactions between human communities and multi pathogens, both within and between specific social and environmental context.

Alignment between the biological modules (as reported in Table 2) and the hierarchical levels was implemented according to previous scheme (as illustrated in Table 3).

Finally, all this information was ordered in a framework diagram for level and scales (as illustrated in Figure 1).

In fact, I-II-III levels contain structural information about viral biology, cell response, and damage in specific body districts, while V-VI-VII levels report descriptive information about clinical phenotypes, epidemiological dynamics, and social restrictions (as illustrated in Figure 1)

Microecosystems and macroecosystems levels report all functional information about direct and indirect interactions among human host, SARS-CoV-2, other pathogens, or other SARS-CoV-2 strains, and environment. (as illustrated in Table 3; Figure 1). The point of view in these two levels is that the crucial aspect: microecosystems correspond to cell/tissue/organ system, while macroecosystems relate to host/community system. These two levels were not associated with any aspect of COVID-19 because of the lack of exhaustive data (as illustrated in Figure 1).

Organically, Table 4 represents the conceptual diagram of the seven hierarchical levels of organization of an infectious disease system related to SARS-CoV-2 infection processes as resulted from the domain-based scoping review, with the associated macroscale and microscale for each level and the types of reciprocal influences among macroscale, microscale, and environmental.

Such model framework can be enlarged with other and current information and detailed by adding new submodules, and it could be represented as a conceptual diagram of the seven hierarchical levels of organization of an infectious disease system, which could be applied also to other infection diseases.

## 4. Discussion

The molecular pathophysiology that links SARS-CoV-2 infection to COVID-19 clinical manifestations is complex and spans multiple biological pathways, cell types, and organs. To gain insights into this complex network, the biomedical research community needs to approach it from a systems perspective, collecting mechanistic knowledge scattered across scientific literature and bioinformatic databases and integrating it using formal systems biology standards.

COVID-19 Disease Map project represents a focal point to organize information about COVID-19 pathogenesis: it is an open-access collection of computational diagrams and models of molecular mechanisms of COVID-19, curated by biocurators, domain experts, modelers, and data analysts. The map is constantly evolving, and it is continuously refined, updated, analyzed, and shared. Currently, this repository reports 41 diagrams containing 1,836 interactions among 5,499 elements, supported by 617 publications and preprints [17]. As part of this important experience, we suggest introducing new interactions into the existing diagrams [16,17].

Despite the increasing knowledge about COVID-19, there are many aspects still unclear and in need of further multiomics investigations, such as the pathophysiological pathways perturbed under comorbidities’ conditions and the degrees of severity.

The virus–host interactome is a network of virus–human protein–protein interactions (PPIs) that can help understanding COVID-19 mechanisms. It can be expanded by merging virus-host PPI data with human PPI and protein data to discover clusters of interactions indicating human mechanisms and pathways affected by SARS-CoV-2 [11,16].

Combined omics technologies could significantly contribute to improve the current understanding of COVID-19 pathology, as reported in our previous review on multiomics COVID-19 studies. However, the enormous amount of information available in the models, still needs to be integrated and harmonized. Thus, the development of disease models must rely on an active involvement and interpretation of domain experts.

Based on the above considerations, our modular design of conceptual disease model was built in analogy to the framework of two studies, chosen and evaluated by interdisciplinary working groups [19].

In the Table 2 are reported the key concepts of the framework and modular logic of a biological COVID-19 model. The modular design of this conceptual model framework was compared to the results of the domain-based scoping review (as reported in Table 1), finding an almost complete overlap and a direct correspondence between module and domain.

This COVID-19 model framework was inspired by concept of infectious disease model system proposed by Garira. This theory considers the extension of the relativity principle in physics to the dynamic of the infectious diseases systems (“replication-transmission relativity theory”) and provides scientific basis for a systems level description of infectious diseases using multiscale modeling methods.

The Garira model allows to design every infectious disease as a multilevel and multiscale system organized into seven main hierarchical levels [22]. In our work, we verified that the framework of the COVID-19 conceptual model is adaptable to Garira model. We also verified that in the model framework that was built, there is no privileged/absolute scale determining disease dynamics, and we identified only interactions among microscale, macroscale, and type of environmentally transmitted infections.

Such structural and functional information about cell response against virus and tissue/organ damages, as well as description of clinical phenotypes, epidemiological dynamics, and social restrictions are the scaffold to apply computation and mathematical model on biological and epidemiological systems [23,24,25,26].

We designed a conceptual diagram of the seven hierarchical levels, and the types of reciprocal influences between macroscale, microscale, and environment in relation to SARS-CoV-2 infection processes.

Finally, this model framework adapted and modified for COVID-19, allows a correlation among host, pathogen, and environment, developing a quantitative evaluation at different scales of the complex multiple biological pathways involved at different levels (cells, tissues, organs, etc.). From this point of view, the results of the scoping review represent the first experimental confirmation of this model, and otherwise, the model can be considered as validated by these results. Both the conceptual model framework and domain-based scoping review constitute a first operational result within an overall research project (i.e., It-IDRIN Project) whose main objective is an aggregation of clinical structures with “omics” competences in a collaborative network focused on pathology models.

In this context, although omics data could help to fill this model framework, providing signatures and pathways form specific phenotypes, they can give only a structural view, limited spatially and timely. Consequently, this model could be useful in research activities (experimental studies), finalizing it to design adaptive trails.

Thus, a network model of molecular interactions, based on omics data, can identify specific mechanisms of host–pathogen interactions, finding the degree of coherence in interactome with the hierarchical structure of the model. This computational approach could define whether an interaction is real, determining the molecular level involved, and correlating the cell/tissue/organ level involved.

Model simulations can help investigate a complete biological process instead of considering smaller segments or aspects, detail a segment of a process or simplify a very large one, suggest or even direct future experiments, and predict the behavior of a system under given conditions.

## 5. Conclusions

The development of disease model framework relies on an active involvement of domain experts. Multiscale modeling of infectious diseases aims to characterize the complexity of infectious disease systems.

The conclusive result is a methodology to design multiscale models of an infectious disease complex, integrating different kinds of data. This methodology is based on implementing a three-stage strategy in the research and development process for multiscale models of infectious disease systems. Further, such methodology could be applicable (with minor modifications) to multiscale modeling of other structurally organized complex systems beyond infectious disease systems.

This research and development process for multiscale models cannot be considered unique, complete, and final. Probably, it is bound to be improved, but it constitutes a good starting point, which may be useful as a basis for further refinement.

## Figures and Tables

**Figure 1:** Diagram of seven main hierarchical levels of organization of an infectious disease system applied to COVID-19. For each level, scales were reported, along with biological and pathological mechanisms and epidemiological data.

**Table 1:** Scoping review: multiomics approach and domains identification literature based. In columns the conceptual sub setting, descried in Montaldo and colleagues, are reported: domain groups, wide conceptual category; domain, subdomain, and function (in bold and underlined, black dot and empty dot, respectively); scale of domain.

Domain Groups	Network-Domains/Subdomains	Scale/Domains
**Virus**	**Molecular characterization** Viral genomics ◦ Genome evolution ◦ Genome hotspots for mutation ◦ Intrahost variability Viral proteomics ◦ Single viral protein ◦ Whole viral proteome Virus–Host interactions ◦ RNA-protein inter. ◦ Virus - host PPIs	Cell Microenvironment
	**Mechanism of entry/viral proteins** Entry factor human tissues Virus–Host Receptor Interact	
**Pathways**	**Pathway** Signal transduction Translation and post translation modifications Immune system ◦ Innate ◦ Adaptive Cell damages Main pathways ◦ Complement activation-coagulation ◦ Inflammation ◦ Oxidative Pathways ◦ Metabolism (lipid, amino acid, fatty acid)	Tissue Organ
	**Host signatures** Soluble mediators Immune response ◦ lung and other tissues ◦ peripheral blood ◦ specific cell types in blood immune cells	
**Phenotype**	**Phenotypes** Comorbidities not sharing COVID-19 pathogenesis Comorbidities associated a related COVID-19 pathways	Organism Macroenvironment
	**Outcome** Severity related to DEG *, DEP ** analysis in: ◦ Lung ◦ Other organs and tissues ◦ Immune response	

* Differentially Expressed Genes; ** Differentially Expressed Proteins.

**Table 2:** COVID-19 model biological keys based framework and modular logic. * Submodels and Figure S1. and garnered by scoping review of Montando and colleagues.

Module	Submodule/Functions *
A. Cell infection and viral replication	1. Tissue microenvironment cell membrane contact (virions travel in the tissue microenvironment to reach a cell membrane): passive transport target cell type and site
	2. Binding receptor on the cell’s membrane (ACE2 system)
	3. Endocytosis process
	4. Viral replication copying and translate viral RNA synthesis viral proteins.
	5. Assembled virions exported from the cell by exocytosis.
**Module**	**Submodule/Functions**
B. Infected cell response	1. Activation IFN type 1 signal to control and to slow viral replication to activate an inflammatory response, and induces apoptosis activators and regulators of the innate and adaptive immune response inhibiting IFN production and suppressing IFN signaling (non-structural proteins produced by SARS-CoV-2).
	2. Cell death process Apoptosis Necroptosis Pyroptosis
**Module**	**Submodule/Functions**
C. Inflammatory and immune responses	1. Pneumocytes and alveolar macrophages SARS-CoV-2 replication in pneumocytes and alveolar macrophages timing of IFN activation
	2. Innate immune response macrophages and neutrophils T cell infection (direct cytopathic effect of the virus), decreased numbers of T cells, functional exhaustion of natural killer (NK) cells Excess IFN secretion, recruitment inflammatory cells (macrophages and neutrophils)
	3. Endothelial damage local and systemic Lung dysfunction related to high levels of IFN-α,β, increased macrophage and neutrophil presence Delayed IFN-α,β production also promotes inflammatory macrophage recruitment activated macrophages also produce other proinflammatory cytokines like IL-1, IL-6, and TNF-α The excess production of IL-1 and IL-6 related to several viral proteins shown to directly activate the inflammasome pathway
	4. Tissue damage and cytokines acute respiratory distress due to reduced tissue integrity, further immune infiltration, fluid leakage and edema induced extensive tissue damage by proinflammatory cytokines (e.g., IL-2, IL-7, IL-10, G-CSF, IP-10, MCP-1, MIP-1A, and TNF-α
**Module**	**Submodule/Functions**
D. Inflammatory and clinical outcome (phenotypes)	1. Dysregulated /amplified immune response and chemokines: replication in the lower airways persistence
	2. Systemic disease: interactions of viral infection, cytokine production, immune response Pre-existing diseases (diabetes, hypertension, immune diseases, obesity) Without comorbidity
	3. Clinical syndromes: hemophagocytosis, intravascular coagulation, ARDS, organ failure Pre-existing diseases (diabetes, hypertension, immune diseases, obesity) Without comorbidity

**Table 3:** Alignment between biological modules and hierarchical levels. Submodules were posed in macroscale/microscale.

	Host		Pathogen	
Hierarchical Levels (*)	**Microscale** **(within)**	**Macroscale** **(between)**	**Microscale** **(within)**	**Macroscale** **(between)**
I cell Module A, B	A2, B1, B2	A1, B1, B2	A4, A5	A3, A4
II tissue Module C	C1, C2	C3, C4		
III organ/anatomical compartment Module C	C3	C4, D1		
IV microecosystems Modules C + B + A	Modules A, B, C	Modules A, B, C		
V host organism Module D, A	D3, A2	Transmission risk in hospital and family; social distancing		
VI community	Epidemiologic enquires (familiar and hospital cluster) and contact tracing, restriction policies	Global surveillance against COVID-19 and restriction traveling		
VII macroecosystems	Contribution of V-VI- VII levels	Contribution of V-VI- VII levels		

(*) hierarchical levels in descending order, from VII to I level.

**Table 4:** Conceptual diagram of the seven hierarchical levels of organization of an infectious disease system and associated macroscale and microscale. Types of reciprocal influences between macroscale, microscale, and environment related to SARS-CoV-2 infection processes. Free adapted and modified from Garira (2020).

	Hierarchical Levels Macro/Micro Hierarchy in Descending order from VII to I Level	Description	Influence Macroscale/Microscale, Type I, II *
			Environmental Infl. Type A,B,C **
	VII The macroecosystem level within-macroecosystem (microscale) between-macroecosystem (macroscale)	the different host (humans, animals) and communities (national, regional, local, …) are considered as ecosystems. The microscale and macroscale for this level of organization of an infectious disease system are the within-macroecosystem scale and the between-macroecosystem scale respectively.	Type II C
	VI The community level within-community (microscale) between-community (macroscale)	level described in terms of single pathogen species/strain as well as single host species and multiple communities. The microscale and macroscale are the within-community scale and the between-community scale.	Type I B
	V The host/organism level within-host (microscale) between-host (macroscale)	level described in terms of single pathogen species/strain as well as single host species and single community. The level has the within-host scale and between-host scale as its microscale and macroscale respectively. The form of reciprocal influence consists of both superinfection, that is, repeated infection before the host recovers from an infectious episode (for the influence of between-host scale on within-host scale) and pathogen excretion/ shedding (for the influence of within-host scale on between-host scale).	Type II B
	IV The microecosystem level within-microecosystem (microscale) between-microecosystem (macroscale)	level described in terms of multiple organs/anatomical compartments and multiple pathogen strains replication. The different organs/anatomical compartments (lung, gut, kidney, heart, stomach, liver, skin, blood, etc.) are considered as ecosystems. The microscale and macroscale are the within-microecosystem scale and the between-microecosystem scale respectively. At this level, ecological process/ interactions influence infectious disease dynamics, which include the competitive species/strains interactions and the mutualistic interactions between the multiple pathogen species/strains.	Type I B
	III The organ/anatomical compartment level within-organ compartment (microscale) between-organ compartment (macroscale)	level described in terms of single pathogen /strain and multiple organs/anatomical compartments (lung, brain, gut, kidney, muscle, heart, pancreas, stomach, liver, spleen, bone, adrenal, skin, adipose, and blood). The microscale and macroscale for this are the within-organ/anatomical compartment scale and the between-organ/anatomical compartment scale.	Type I B
	II The tissue level within-tissue (microscale) between-tissue (macroscale)	Different types of tissues (airway epithelium, endothelial epithelium, immune system, …) can be considered in the multiscale dynamics of COVID-19 systems including inflammation, coagulation, and fibrosis. This level has the within-tissue scale and between-tissue scale as its microscale and macroscale respectively	Type I B
	I The cell level within-cell (microscale) between-cell (macroscale)	When integrating the within-cell scale and between-cell scale, different types of target cells can be considered in the multiscale dynamics of infectious disease dynamics such: pneumocytes, alveolar macrophages, CD8+T, CD4+ T. This level has the within-cell scale and between-cell scale as its microscale and macroscale respectively.	Type I B

* Macro-micro-scale mutual influence. Type I: the microscale influences the macroscale. Type II: the macroscale influences the microscale; ** Environmental influence: Type A: there is no pathogen replication at the microscale (within-host scale). Type B: the pathogen only replicates at the microscale (within-host scale). Type C: the pathogen replicates at both microscale (within-host scale) and macroscale (between-host scale).

## Data Availability

The data used to fill out this framework is reported in Table S1.

## Supplementary Materials

The following are available online at https://www.mdpi.com/article/10.3390/v13071309/s1, Table S1: key concepts, obtained by scoping review in Montaldo and colleagues, for the framework of a biological COVID-19 model. References [3,4,5,6,16,19,20,21,22,27,28,29,30,31,32,33] are cited in the Supplementary Materials.
